The article "Tspan8 and Tspan8/CD151 knockout mice unravel the contribution of tumor and host exosomes to tumor progression" was retracted in 2025. Reasons: unreliable data; lack of ethics approval or compliance; concerns about the data; concerns about the images.

# Tspan8 and Tspan8/CD151 knockout mice unravel the contribution of tumor and host exosomes to tumor progression

**DOI:** 10.1186/s13046-018-0961-6

**Published:** 2018-12-12

**Authors:** Kun Zhao, Zhe Wang, Thilo Hackert, Claudia Pitzer, Margot Zöller

**Affiliations:** 1 Pancreas Section, University Hospital of Surgery, Ruprecht-Karls-University, Heidelberg, Germany; 2 Interdisciplinary Neurobehavioral Core, Institute of Pharmacology, Ruprecht-Karls-University, Heidelberg, Germany; 3 Present Address: Department of Oncology, First Affiliated Hospital of Guangdong Pharmaceutical University, Guangdong, China

**Keywords:** Tspan8 knockout, CD151 knockout, Exosomes, Metastasis, Angiogenesis, Hematopoiesis

## Abstract

**Background:**

The tetraspanins Tspan8 and CD151 promote metastasis, exosomes (Exo) being suggested to be important in the crosstalk between tumor and host. The contribution of Tspan8 and CD151 to host versus tumor-derived exosome (TEX) activities being not defined, we approached the questions using 3-methylcholanthrene-induced (MCA) tumors from wt, Tspan8ko, CD151ko and Tspan8/CD151 (db)ko mice, implanted into tetraspanin-competent and deficient hosts.

**Methods:**

Tumor growth and dissemination, hematopoiesis and angiogenesis were surveyed in wild type (wt), Tspan8ko, CD151ko and dbko mice bearing tetraspanin-competent and -deficient MCA tumors. In vitro studies using tumor cells, bone marrow cells (BMC) and endothelial cells (EC) elaborated the mechanism of serum (s)Exo- and TEX-induced target modulation.

**Results:**

Tumors grew in autochthonous and syngeneic hosts differing in Tspan8- and/or CD151-competence. However, Tspan8ko- and/or CD151ko-tumor cell dissemination and settlement in metastatic organs was significantly reduced in the autochthonous host, and less severely in the wt-host. Impaired wt-MCA tumor dissemination in the ko-host confirmed a contribution of host- and tumor-Tspan8/-CD151 to tumor cell dissemination, delivery of sExo and TEX being severely impaired by a Tspan8ko/CD151ko. Coculturing tumor cells, BMC and EC with sExo and TEX revealed minor defects in epithelial mesenchymal transition and apoptosis resistance of ko tumors. Strongly reduced migratory and invasive capacity of Tspan8ko/CD151ko-MCA relies on distorted associations with integrins and CAM and missing Tspan8/CD151-promoted recruitment of proteases. The defects, differing between Tspan8ko- and CD151ko-MCA, were rescued by wt-TEX and, less efficiently Tspan8ko- and CD151ko-TEX. Minor defects in hematopoietic progenitor maturation were based on the missing association of hematopoietic growth factors /− receptors with CD151 and, less pronounced, Tspan8. Rescue of impaired angiogenesis in ko mice by wt-sExo and promotion of angiogenesis by TEX depended on the association of Tspan8 and CD151 with GPCR and RTK in EC and tumor cells.

**Conclusions:**

Tspan8-/CD151-TEX play central roles in tumor progression. Tspan8-/CD151-sExo and TEX contribute by stimulating angiogenesis. Tspan8 and CD151 fulfill these tasks by associating with function-relevant proteins, the additive impact of Tspan8 and CD151 relying on differences in preferred associations. The distinct Tspan8 and CD151 contributions suggest a blockade of TEX-Tspan8 and -CD151 promising for therapeutic intervention.

**Electronic supplementary material:**

The online version of this article (10.1186/s13046-018-0961-6) contains supplementary material, which is available to authorized users.

## Background

Tumor progression depends on the crosstalk with the host promoting angiogenesis, tumor cell migration and settlement in distant organs [1]. Tumor cells support these processes via provision of exosomes (Exo), which deliver angiogenesis stimulating factors, chemokines, chemokine receptors, adhesion molecules and proteases [2–5].

Exosomes, small vesicles delivered by many cells and abundantly by tumor cells [6], are composed of a lipid bilayer with incorporated and attached membrane molecules. The small Exo cytoplasm contains cytosolic proteins, coding and noncoding RNA and DNA [7]. Exo distribute through the body, selectively bind to or fuse with target cells or are uptaken [8, 9]. All Exo components being function-competent [10, 11], binding/uptake is accompanied by target modulation [3–5, 12]. Finally, cells deliver several types of Exo [9] that differ by early endosome (EE) origin from cytoplasmic organelles or invaginated membrane domains, like caveolae, clathrin-coated pits [11, 13] or tetraspanin-enriched microdomains (TEM) characterized, besides others, by distinct lipid composition [14, 15]. Notably, tetraspanins are the only consistently enriched protein family in Exo [9].

Tetraspanins are highly conserved 4-transmembrane proteins with a small and a large extracellular loop [16]. The latter accounts for dimerization and association with non-tetraspanin transmembrane partner molecules [17]. Besides few direct protein-protein interactions, and due to the lipid composition of TEM, tetraspanins are characterized by a multitude of attached proteins, including integrins, CAMs, RTK, proteases, cytoskeleton and cytosolic signal transduction molecules [18–20]. Tetraspanins mostly acting as molecular facilitators via the associated proteins, it is important that tetraspanin webs are maintained during TEM invagination and vesicle trafficking and are recovered in the released Exo [21].

The tetraspanins CD151 and Tspan8 promote tumor cell dissemination and metastasis [22, 23]. CD151 contributes to pericellular MMP activation allowing for focal ECM proteolysis [20] and influences MMP expression and colocalization at the leading edge [24, 25]. CD151 also is engaged in focalizing laminin (LN)-binding α3β1 and α6β4, migration / invasion being strengthened by α3β1 co-internalization [22, 26]. The association with growth factor/chemokine receptors stimulates downstream signaling activation [27] promoting carcinogenesis and metastasis [28–30]. CD151 also supports angiogenesis. By recruiting CD151, LN1-bound α6β1 stimulates embryonic stem cell differentiation into endothelial cells (EC) [31]. High Tspan8 expression promotes hepatocellular carcinoma lung metastases [32, 33] and ovarian cancer invasion [34]. Glioblastoma migration and drug resistance rely on Tspan8 complex formation and FAK activation [35]. Tspan8 complexes with α3 and rictor, a key component of the mTORC2 complex, supports migration [36]. A contribution of Tspan8 to metastasis was confirmed by anti-Tspan8 inhibiting colon cancer growth in vivo, without affecting proliferation and apoptosis resistance in vitro, which points towards Tspan8 / Tspan8-complexes responding to environmental signals [37]. According to the TEM-derived biogenesis, Exo-Tspan8 and -CD151 act in concert with associated molecules. Thus, tumor Exo (TEX) Tspan8-α4β1 induce disseminated intravascular coagulation as a sequel of overshooting angiogenesis [38]. On the other hand, Tspan8-α6β4 TEX promote migration and metastasis [39], also described for CD151-TEX [40].

Taken together, there is increasing evidence that the engagement of CD151 and Tspan8 in tumor progression and angiogenesis relies on the crosstalk between targets and Tspan8+ / CD151+ Exo [21]. This assumption can be controlled by implanting tetraspanin-competent and -deficient tumors into wt hosts. Tumor implantation into tetraspanin-ko hosts additionally allows to judge on a host-derived Tspan8+ / CD151+ Exo contribution to tumor progression. As previous work using Tspan8ko, CD151ko and Tspan8ko/CD151ko (dbko) mice indicated an additive engagement of CD151 and Tspan8 in angiogenesis and keratinocyte migration, dbko MCA tumors and dbko mice were included [41]. The analysis of autochthonous and syngeneic tumors differing in Tspan8 and/or CD151 competence confirmed the importance of Tspan8 and CD151 in Exo biogenesis and Exo target binding. Furthermore, Tspan8 and CD151 TEX show partially supplementing engagement in tumor cell dissemination, distant organ settlement and angiogenesis. Host tetraspanin-competent Exo contribute to tumor cell settlement in the bone marrow and angiogenesis.

## Methods

### Mice and tumors

C57BL6 Tspan8ko, CD151ko and Tspan8ko/CD151ko (dbko) mice and MCA-induced tumors in wt C57BL6 and the ko mice are described [41, 42]. Homozygosis was controlled by genotyping (Primers: Additional file 1: Table S1) [41, 42]. Tumors were maintained in RPMI1640/10%FCS/antibiotics/glutamine and IGS supplement (Sigma).

### Antibodies and chemicals: Additional file 1: Table S2

#### Tissue collection

Solid organs and lymph nodes (LN) were shock frozen or dispersed by meshing through fine gauze. Bone marrow cells (BMC) were collected by flushing femora and tibiae with PBS, peripheral blood leukocytes (PBL) was collected by heart puncture using heparinized syringes, isolating PBL by Ficoll/Hypaque centrifugation.

#### Exosome preparation

sExo/TEX preparation and SP-Dio_18_(3)-labeling followed described protocols [15], modified by 0.22 μm filtration of cleared supernatants.

#### Sucrose density gradient centrifugation of cell lysates

Cell lysates in 2.5 M sucrose were overlaid by a discontinuous sucrose gradient (0.25 M–2 M) and centrifuged (15 h, 150,000 g), collecting twelve 1 ml fractions.

#### Immunoprecipitation (IP), Western blot (WB)

Cells were lysed in HEPES buffer/1%Lubrol/1 mM PMSF/1 mM NaVO_4_/10 mM NaF/protease inhibitor mix (30 min, 4 °C), mild lysis conditions were used for not destroying loosely attached protein complexes. Lysates were centrifuged (13,000 g, 10 min, 4 °C), mixed with antibody (1 h, 4 °C) and incubated with ProteinG-Sepharose (1 h). Washed and dissolved complexes/lysates were resolved on 10–12% SDS-PAGE, developing blots with ECL after transfer, blocking and blotting.

#### Zymography

Culture supernatant of MCA tumors, starved for 24 h, was centrifuged (15 min, 15,000 g). Aliquots, incubated with Laemmli buffer (15 min, 37 °C), were separated in a 10% acrylamide gel containing 1 mg/ml gelatin. Washed gels (2.5%Triton) were incubated in developing buffer (37 °C, 48 h) and stained with Coomassie-blue.

#### Adhesion

Cells were seeded on BSA-, collagen (coll)-, laminin (LN)-, or fibronectin (FN)-coated 24w-plates. After adhesion (2 h, 37 °C, 5%CO_2_) and washing, adherent cells were stained with crystal-violet, determining optical density at 595 nm. Adhesion (triplicates) is presented as % input cells.

#### Migration

Cells in the upper part of a Boyden chamber (RPMI/0.1%BSA) were separated from the lower part (RPMI/20%FCS) by 8 μm pore size polycarbonate-membranes. After 16 h the lower membrane side was stained (crystal-violet), measuring OD595 after lysis. Migration (triplicates) is presented as % input cells. In an in vitro wound healing assay, a subconfluent monolayer was scratched with a pipette tip. Wound closure was controlled by light microscopy.

#### Invasion

Polycarbonate membranes (8 μm pore size) transwell permeable supports were coated with 100 μl 1:5 diluted Matrigel and kept in a humidified atmosphere (37 °C, overnight). After washing, 5 × 10^4^ cells in 200 μl RPMI/1%BSA were placed on the gels. The lower chamber contained RPMI/20%FCS. After 48 h (37 °C, 5%CO_2_), cells not invading the gels were washed-off. Matrix invasion and recovery on the lower membrane side was evaluated microscopically and photometrically after crystal-violet staining and lysis.

#### Soft agar assay

Tumor cells in 0.3% agar were seeded in 6-well plates on a preformed 1% agar layer, counting colonies after 3wk.

#### Proliferation

Cells (2 × 10^4^) were seeded in F-bottom 96-well plates adding after 48 h ^3^H-thymidine (10 μCi/ml), evaluating ^3^H-thymidine incorporation after 16 h (β-counter).

#### Apoptosis

Cells (1 × 10^5^) were grown for 48 h in RPMI/10%FCS containing cisplatin. Survival was monitored by flow-cytometry after annexinV-APC/PI staining or by the MTT assay or by ^3^H-thymidine uptake.

Flow-cytometry: TEX/sExo (10 μg) were coupled to 1 μl Latex beads (LB). After blocking (100 mM glycine) and washing, TEX/sExo-loaded LB were stained using the same standard protocol as for cells. For intracellular staining, cells/LB-coated TEX/sExo were fixed and permeabilized in advance. Samples were analyzed in a FACSCalibur using the CellQuest program.

#### Histology

Snap frozen sections (8 μm) were fixed, incubated with antibodies, washed, exposed to biotinylated secondary antibodies and alkaline phosphatase conjugated avidin-biotin solution. Sections were counter-stained with hematoxilin. Digitized images were generated using a Leica DMRBE microscope.

#### Confocal microscopy

Cells were fixed, permeabilized, blocked, incubated with primary antibody, washed, incubated with Cy2-conjugated secondary antibody and after washing and blocking stained with an additional primary antibody and a Cy3-conjugated secondary antibody. Slides were mounted in Elvanol. Digitized images were generated using a Leica LMS800 microscope and the Carl Zeiss Vision software for evaluation.

#### In vivo assays

Mice received a subcutaneous (sc) application of 2 × 10^6^ MCA tumor cells. Tumor growth was monitored weekly. Mice were sacrificed when the local tumor reached a mean diameter of 1.5 cm or latest after 240d. Mice were controlled for visible metastases. Blood, LN, bone marrow, liver and lung were collected and cultured controlling for latent tumor cell outgrowth. Animal experiments were Government-approved (Baden-Wuerttemberg, Germany) and carried out in accordance with EU Directive 2010/63/EU.

#### Statistics

*P* values < 0.05 (in vitro: two-tailed Student’s t-test, in vivo: Kruskal-Wallis test after Bonferroni Holm correction, where indicated) were considered significant.

## Results

### Characterization of wt, Tspan8ko and/or CD151ko MCA-tumors, endothelial cells, bone marrow cells, TEX and serum exosomes

Exploring a possible impact of host Exo and TEX Tspan8 and CD151 on tumor growth and progression required a criss-cross evaluation of the MCA wt, Tspan8ko and/or CD151ko tumors in the autochthonous and the syngeneic host differing in Tspan8 and/or CD151 competence. Awareness of cell and Exo/TEX Tspan8- and CD151-dependent changes in the protein profile being a prerequisite for the interpretation of in vivo and functional in vitro studies, these data are summarized for tumor cells / TEX, EC, BMC and sExo in Additional file 1: Figure S1.

Tetraspanin expression of MCA tumors was evaluated by flow-cytometry and WB. The tumors express CD9 at a high, CD63 and CD81 at a rather low level, mean level CD151 expression is abolished in CD151ko- and dbko-MCA tumors and low level Tspan8 expression in Tspan8ko- and dbko-MCA tumors (Additional file 1: Figure S1a, c). Characterization of the TEX protein profile became important as one route of Exo biogenesis proceeds via TEM internalization, trafficking of the originating EE involving tetraspanins [13, 43]. TEX express CD9, CD151 and Tspan8 at a higher level than cells (Additional file 1: Figure S1b, c).

MCA tumors express the tumor markers CD24, S100A4, CD184, TGFβ1, CD138, thrombospondin (ThbSp) and tissue factor (TF) at high to medium and ALDH1/2, CD133, HSP70 and HSP90 at low level. Expression does not significantly differ between wt- and ko-MCA lines (Additional file 1: Figure S1d). Expression of the tumor markers HSP70 and HSP90 was significantly higher in TEX than cells. Ko-TEX differed by slightly reduced ThbSp recovery (Additional file 1: Figure S1e). Similar findings accounting for several ko-MCA-tumors (data not shown), we proceeded with these lines.

The higher expression of tetraspanins and HSPs in Exo being known [9], only ThbSp recruitment into ko TEX was impaired.

Tetraspanins acting as molecular facilitators of associated molecules, the impact of Tspan8 and CD151 on adhesion molecule, protease and signaling receptor expression required exploration.

The MCA cells highly express CD44, CD29 and CD49f. Expression of CD49f is slightly reduced in ko-MCA cells, low CD49c and CD62L expression is reduced in Tspan8ko−/dbko- and CD56 and CD106 in CD151ko−/dbko-MCA (Additional file 1: Figure S1f, h), reduced expression being also seen in ko-TEX. The most impressive changes in TEX were increased recovery of several integrins, CAMs and selectins. Reduced CD49c in Tspan8ko- and CD56 and CD106 expression in CD151ko-MCA cells and -TEX (Additional file 1: Figure S1f-h) points towards a linkage of CD49c to Tspan8 and of CD56 and CD106 to CD151.

Flow-cytometry and WB revealed high MMP2, MMP3, uPA and ADAM10 and medium to low uPAR, MMP9, MMP14 and TACE expression in wt-MCA cells. UPAR, uPA, MMP2 and MMP3 expression was reduced in Tspan8ko−/dbko-, TACE expression was reduced in CD151ko/dbko, MMP9, MMP14 and ADAM10 expression was reduced in all 3 ko-MCA lines. Except for a strong increase in uPAR, the protease expression profile of MCA-TEX resembled that of cells (Additional file 1: Figure S1i-k).

Tetraspanins cooperate with RTK [44]. High TGFβRI, -II and VEGFR2 expression was reduced in the three ko lines. PDGFRB, VEGFR3 and EphA4 expression was only reduced in Tspan8ko MCA (Additional file 1: Figure S1 l).

EMT and apoptosis-resistance are important tumor parameters. Both epithelial E- and mesenchymal N-cadh were expressed at a high level irrespective of a Tspan8ko and/or a CD151ko. FN and vim expression are low, FN expression being reduced in CD151ko-MCA cells. Only the EMT-related transcription factors Nanog and slightly NOTCH expression was reduced in the three ko lines and FOXO3 and Frizzled expression in CD151ko cells (Additional file 1: Figure S1 m). Low death receptor expression was not affected by a Tspan8ko and/or a CD151ko. BAD phosphorylation and BclXl expression was slightly reduced in Tspan8ko cells, but proapoptotic BAX expression was not affected. Unexpectedly, Casp3 and cleaved Casp9 expression was slightly reduced in Tspan8ko cells, but not TEX (Additional file 1: Figure S1n, o).

Finally, a Tspan8ko did not affect the sExo profile and in CD151ko- and dbko-mice only CD54 expression was reduced. Thrombocyte markers (CD41, CD61) were unaffected (Additional file 1: Figure S1p).

BMC and EC were selected as non-transformed cells. Tumor growth depends on angiogenesis [5], which involves tetraspanins [45–49]. Tumor progression frequently is accompanied by anemia and deviation of hematopoiesis towards immunosuppressive components. The bone marrow also is a preferred metastatic organ.

BMC were characterized by flow-cytometry for tetraspanin, progenitor marker, hematopoietic chemokine and -receptor expression. There was a slight reduction in CD9 expression in BMC of the 3 ko-mice, CD63 expression was reduced in CD151ko- and dbko-BMC. KIT, CD34, CD62P, TER119 and Gr1 expression was reduced in all 3 ko-BMC; CD44 expression was only slightly reduced in CD151ko- and dbko-BMC. OPN expression was reduced in the 3 ko lines, CXCL10 and MCSFR expression was more strongly affected in CD151ko−/dbko-BMC. In brief, Tspan8 and CD151 possibly affect early hematopoietic progenitors, erythropoiesis and thrombopoiesis. (Additional file 1: Figure S1q).

Tetraspanin expression was not affected in EC-enriched cells, CD31 and CD34 EC marker expression was slightly reduced in Tspan8ko−/dbko-EC, CD106 and CD62P in CD151ko−/dbko-EC. OPN, VEGFR2 and EphA4 were reduced in all 3 ko-EC and SDF1 in CD151ko−/dbko-EC (Additional file 1: Figure S1r). These findings would be in line with a minor impact of Tspan8 and CD151 on EC progenitor maturation, but impaired EC activation and proliferation.

Briefly, a Tspan8ko and/or a CD151ko only affect expression of selected markers and the impact is minor. In most instances the response to a Tspan8ko and a CD151ko differed and was stronger in dbko cells, which we interpret towards a partially additive Tspan8 and CD151 contribution. Exosomes mostly reflect the changes in the cellular protein profile. However, in some instances differences between the Tspan8ko and the CD151ko became hidden that may relate to the pool of Exo deriving from distinct biogenesis pathways.

### Tspan8- and CD151-dependent exosome delivery and binding

Exo biogenesis can proceed via TEM internalization and Exo use tetraspanin complexes for binding [15, 40]. Thus, Tspan8 and CD151 may affect sExo / TEX delivery and target binding.

First to note, ko-MCA secrete significantly less TEX than wt-MCA (Additional file 1: Figure S2a) and fewer sExo are recovered from ko- than wt-mice (Additional file 1: Figure S2b). Wt-, Tspan8ko- and CD151ko-sExo and -TEX uptake by Tspan8ko- and CD151ko-MCA is not distorted. Instead, dbko-sExo and -TEX are poorly taken-up by wt- and ko-MCA, examples being shown for the uptake of TEX by CD9+ MCA cells (Additional file 1: Figure S2c, d).

Reduced dbko-sExo and -TEX uptake also accounts for EC, where Tspan8ko- and CD151ko-sExo uptake was additionally impaired (Additional file 1: Figure S2e). Instead, mostly CD151ko- and dbko-BMC displayed reduced sExo/TEX uptake (Additional file 1: Figure S2f). Wondering whether this accounts for subpopulations, unseparated BMC were incubated with Dio-labeled wt-sExo and -TEX and stained for selected markers. The analysis confirmed reduced recovery of KIT+ and TER119+ and, less pronounced, Gr1+ Tspan8ko-, CD151ko- and dbko-BMC, the percent of wt-sExo/−TEX positive BMC being correspondingly decreased (Additional file 1: Figure S2 g). Presenting the data as relative percent of sExo+/TEX+ BMC revealed two informations. First, Gr1+ and CD11b + BMC take-up sExo/TEX more avidly than KIT+ and TER119+ cells. Furthermore, KIT+ cells take-up TEX more readily than sExo (Additional file 1: Figure S2 h).

The findings imply a strong impact of CD151 and Tspan8 on sExo and TEX delivery. In addition, sExo/TEX-Tspan8 and -CD151 contribute to target binding/uptake. As only the uptake of dbko-sExo and -TEX was consistently affected, we suggest that sExo/TEX-Tspan8 and -CD151 may mutually replace. The weaker effects of dbko-sExo/TEX uptake by BMC and EC point towards distinct tetraspanins, possibly CD9, CD63 or CD81, being additionally engaged in uptake by BMC and EC.

Uptake of sExo may provide a continuous modulator and uptake of TEX may account for reprogramming towards facilitating angiogenesis, tumor cell dissemination and settlement and/or for creating an immunosuppressive milieu [50–53]. Tetraspanins being engaged in Exo biogenesis and targeting and coordinating associated molecules’ activity, we expected unraveling a unifying concept by evaluating the tetraspanin contribution, monitored for Tspan8 and CD151 in MCA tumors, BMC and EC.

### Tumor growth in wt- and ko-mice

Whether host Tspan8 and CD151 affect tumor growth, was controlled by sc injection of wt- and ko-MCA-tumors into wt- and ko-mice. The growth rate differs for the 4 MCA lines. The dbko-MCA tumor growing faster, tumor growth could only be compared for the individual tumors in wt- versus ko-mice. Wt-MCA-tumor growth was not affected in CD151ko- compared to wt-mice, but was delayed in Tspan8ko- and dbko-mice. Growth of slowly developing Tspan8ko-MCA tumors was further delayed in dbko-mice. The growth of CD151ko-MCA tumors was retarded in CD151ko- and dbko-mice, the growth of dbko-MCA tumors was delayed in all 3 ko-strains (Fig. 1a, b). The strongest retardation being seen in wt-MCA growth in Tspan8ko and dbko mice was a first indication of host sExo supporting tumor growth. This suggestion was strengthened by evaluating tumor cell dissemination, which strongly differed between wt and ko hosts, but also between wt and ko tumors. Tumor cell outgrowth was evaluated in PB, LN, BM, lung and liver after in vitro culture. Wt MCA cells were regularly recovered in PB, LN, BM, lung and rarely liver. Tumor cell dissemination was particularly affected in Tspan8ko and dbko mice, also apparent by the cumulated tumor cell dissemination. Similar findings accounted for the three ko-MCA lines. Ko-MCA tumors frequently developed LN and lung metastasis in wt-mice, but only in 30–60% of the autochthonous host, the lowest tumor load being observed in dbko-mice. However, the dissemination capacity of the ko MCA tumors was also significantly impaired, when grown in wt-mice, which implies a contribution of Tspan8- and CD151-TEX to dissemination, with a stronger effect of Tspan8 than CD151. Finally, host Tspan8- and CD151-Exo have a distinct impact on dissemination in the blood versus settlement in distinct organs. Dissemination in the blood was most strongly affected in CD151ko-mice, settlement in LN, BM, lung and liver was more strongly impaired in Tspan8ko−/dbko-mice (Fig. 1c).

**Fig. 1:** Tumor growth in Tspan8ko- and/or CD151ko-mice. Wt and ko mice received a sc injection of 2 × 10^6^ wt- or ko-MCA cells. **a** Initiation of tumor growth and mean tumor diameter (6 mice/group); **b** survival and mean survival time of wt- and ko-mice after sc injection of wt- and ko-MCA tumor cells (5 mice/group); *p*-values are indicated; **c** No of mice with migrating tumor cells (PB) and micrometastases in draining LN, BM, lung and liver and mean frequency of mice with disseminated tumor cells per tumor, per mice and per organ; *p*-values (after Bonferroni Holm correction) are indicated; **d** Tabular overview of shock frozen tumor sections (immunohistochemistry) of tetraspanins, adhesion molecules, proteases and angiogenesis-related factors / receptors in wt- and ko-MCA tumors grown in wt and ko mice. Expression was judged as +++: very strong, ++: strong, +: distinct, ±: weak, ±: very weak; **e** immunohistochemistry examples of tetraspanin expression in wt and ko MCA grown in wt and ko mice (scale bar: 100 μm). Tumor growth initiation of wt- and ko-MCA tumors is retarded in ko mice and tumor growth progresses very slowly. Tumor cell dissemination is severely impaired in ko mice, but ko MCA dissemination is promoted in wt mice accompanied by upregulation of adhesion molecules, proteases and angiogenesis markers. Dbko-MCA cells grown in dbko mice were very necrotic. The findings indicate compensatory activities of the host

Flow-cytometry of minced wt-MCA tissue at autopsy showed reduced Tspan8 and VEGFR3 expression in Tspan8ko- and dbko-mice, CD151 expression was reduced in CD151ko- and dbko-mice and VEGFR2 expression was affected in all 3 ko-strains. On the other hand, Tspan8, VEGFR3, Lyve, MMP2 and TGFβ1 expression of Tspan8ko-MCA became increased in wt-mice, but CD106 and VEGFR2 expression was further reduced in CD151ko−/dbko-mice. Finally, CD151 and VEGFR2 expression of CD151ko-MCA was strengthened in wt- and Tspan8ko-mice and VEGFR3 expression in wt-mice (Additional file 1: Figure S3a). The finding suggests that VEGFR3 and MMP2 deficits in Tspan8ko mice and VEGFR2, CD56 and CD106 deficits in CD151ko mice may be partly rescued by wt-sExo.

Immunohistochemistry of shock frozen tumor sections supported the flow-cytometry analysis, where weak expression in the tumor tissue should be taken into account to avoid overestimation of changed expression (Fig. 1d). Slightly reduced CD9 expression in Tspan8ko- and dbko-MCA is increased in wt-mice. Tspan8 expression in wt-MCA becomes reduced in Tspan8ko- and dbko-mice, but Tspan8ko- and dbko-MCA display increased expression in wt-mice. Similar host-dependent changes are seen in CD151 expression (Fig. 1d, e).

Due to the link of tetraspanins with adhesion molecules and proteases [41, 42] their regulation in wt- and ko-hosts became of special interest. CD49c, CD104, CD56 and CD106 expression in wt-MCA was slightly reduced in CD151ko- and dbko-hosts. Lower expression in ko-, particularly CD151ko-MCA was mostly upregulated in the wt-host (Fig. 1d). Wt-MCA MMP9 expression was slightly reduced in ko-mice, but MMP2 and MMP9 expression of Tspan8ko- and dbko-MCA was increased in wt- and CD151ko-mice. MMP2, MMP9 and uPAR expression of dbko-MCA was increased in wt- and single ko-mice (Fig. 1d, Additional file 1: Figure S3b).

VEGFR2, VEGFR3 and Lyve expression in wt-MCA tumors is slightly reduced in ko-mice, but expression of VEGFR3 and Lyve in ko-MCA becomes stronger in wt-mice. CD31+ cells in wt-MCA tumors were reduced in ko-, most strongly CD151ko-mice, but were increased in CD151ko- and dbko-MCA tumors grown in wt-mice (Fig. 1d, Additional file 1: Figure S3c).

Reduced SDF1+ and TF+ cell recovery in wt-MCA tumors grown in ko-mice and rescue of these markers in Tspan8ko- and dbko-MCA tumors, when grown in wt-mice, were most prominent changes in tumor markers (Fig. 1d).

Taken together, host and tumor Tspan8 and CD151 contribute to tumor progression, with only a partial overlap of Tspan8- and CD151-deficits, apparent by the stronger defects of dbko-MCA in dissemination, more strongly impaired angiogenesis of CD151ko MCA and more pronounced deficits in Tspan8ko MCA in distant organ settlement. Flow-cytometry and immunohistology provided first hints towards distinct adhesion molecules, proteases, GPCR and RTK accounting for impaired ko tumor cell dissemination. Furthermore, tumor growth in wt versus ko mice confirmed that wt-sExo can partially cope with ko-MCA deficits. To control these assumptions and to unravel the Tspan8 and CD151 engagement, MCA cells, EC and BMC were cocultured with wt-sExo or wt- and ko-TEX searching for changed functions and hints towards the underlying mechanism.

### Tspan8- and CD151-TEX do not promote apoptosis resistance or a shift towards EMT in MCA tumors

TEX promote high apoptosis resistance of tumor cells [54–56]. The MCA tumors display low apoptosis resistance and the rate of AnnV/PI stained cells did not significantly differ between wt- and ko-MCA tumors after 48 h culture in the presence of cisplatin, confirmed in an MTT assay. However, proliferative activity particularly of dbko-MCA tumors declined more rapidly (Additional file 1: Figure S4a). Addition of wt-TEX, but not ko-TEX promoted proliferative activity of cisplatin-treated (2.5 μCi/ml) Tspan8ko- and CD151ko-, but not dbko-MCA cells (Additional file 1: Figure S4b). Flow cytometry revealed that impaired PI3K/Akt activation of the ko MCA cells became mitigated in the presence of wt-TEX. Concomitantly pBAD and BclXl expression became upregulated (data not shown). The finding argues for an engagement of Tspan8 and CD151 in PI3K/Akt pathway activation. As Tspan8ko and CD151ko MCA equally well responded to wt-TEX treatment, the failure of dbko MCA may rely on poor TEX uptake. Nonetheless, the weak impact exclusively on proliferative activity argues against a Tspan8ko/CD151ko affecting MCA apoptosis resistance.

Tumor cells are characterized by anchorage independent growth and the capacity for EMT, which can initiate or support tumor cell dissemination. Soft agar colony formation of wt MCA was reduced in Tspan8ko- and/or CD151ko-MCA and was partially rescued by wt-TEX (Fig. 3a). Seeding Tspan8ko- and CD151ko-MCA at a low density in medium supplemented with 20 μg/ml wt-TEX, promoted proliferation accompanied by a minor shift towards a more fibroblastoid shape, which was not seen culturing MCA with ko-TEX (Fig. 3b, Additional file 1: Figure S5a, b). The tumor markers ALDH1/2, CD133 and CD24 expression was slightly increased (Additional file 1: Figure S5c). However, reduced FN, FOXO3 and Frizzled expression in CD151ko- and dbko-MCA cells was not or hardly rescued by wt-TEX. Only NOTCH and Nanog expression became restored inTspan8ko- and CD151ko-MCA (Fig. 2c, d). Nanog, NOTCH and Snail also were recovered in the nucleus of wt- and Tspan8ko-MCA and nuclear recovery of Nanog and NOTCH was stronger after wt-TEX treatment of Tspan8ko-MCA (Fig. 2e). But, NOTCH and Nanog also became upregulated by coculture with ko-TEX (Fig. 2f). Thus, TEX slightly promote proliferation and a partial shift towards EMT, which is Tspan8- and CD151-independent.

**Fig. 2:** Anchorage-independent growth, proliferative activity and EMT of wt- and ko-MCA tumor cells. **a** Examples of wt- and ko-MCA cell soft agar colonies in the absence or presence of wt-TEX (30 μg/ml) and mean colony number/1000 cells±SD (3 assays); significant differences between wt and kd cells and between controls and wt-TEX-treated cells are indicated; **b** wt- and CD151ko-MCA cells were seeded at low density in 6-well plates in the absence or presence of wt-TEX. Cell density and morphological appearance were evaluated after 72 h by light microscopy (scale bar: 100 μm); (**c-f**) wt- and ko-MCA tumor cells were cocultured with wt- and ko-TEX for 48 h. **c** Flow-cytometry analysis of EMT marker expression and representative examples; **d** WB of EMT transcription factor expression; **e** WB of EMT transcription factor expression in the cytosol and the nucleus; **f** Flow cytometry analysis of EMT transcription factor expression in Tspan8ko-MCA cells after coculture with wt- or ko-TEX; (**c,f**) mean % stained cells±SD (3 assays); significant differences between wt- and ko-MCA: *, by coculture with TEX: s. Anchorage-independent growth of ko-MCA cells is impaired and partly restored by wt-TEX. Wt-TEX promote a slight shift towards a more fibroid morphology. But, only reduced Nanog and NOTCH expression become upregulated by wt- and ko-TEX without changes in nuclear recruitment. This argues against Nanog and NOTCH upregulation being Tspan8- and CD151-TEX dependent

The minor impact of a Tspan8ko and/or CD151ko on MCA tumorigenic features is in line with unimpaired MCA tumor-induction in the ko-mice. Though with the exception of Nanog and NOTCH, these minor alterations were connected to Tspan8 and CD151, the weak effects unlikely account for the strong impact of a Tspan8ko and a CD151ko on MCA dissemination.

### Tspan8 and CD151, tumor cell adhesion / migration and the impact of TEX

Tspan8 and CD151 preferentially associate with LN-binding integrins, which affects adhesion and motility. Compared to wt-MCA, adhesion of ko-MCA cells to BSA-coated plates was slightly reduced. However, wt-MCA cells poorly adhered to matrix proteins, adhesion of Tspan8ko- and CD151ko-MCA cells being even weaker and dbko-MCA cells did not adhere (Fig. 3a). Distinct to matrix proteins, wt-sExo and -TEX promoted adhesion. Adhesion-supporting activity of Tspan8ko- and CD151ko-TEX was faint and dbko-TEX were inefficient (Fig. 3b).

**Fig. 3:** Adhesion and migration of wt- and ko-MCA tumor cells. **a** Tumor cells were seeded on matrix protein-coated plates. After 4 h incubation and washing, the percent of adherent cells was evaluated by crystal-violet staining measuring OD585; **b** MCA cells were seeded on BSA-coated plates, the medium containing 10% Exo-depleted FCS or 30 μg/ml wt-sExo or -TEX. After 4 h incubation and washing, the percent of adherent cells was evaluated by crystal-violet staining measuring OD585; **a**, **b** mean values±SD (triplicates), significant differences between wt- and ko-cells: *; significant differences between BSA- versus matrix protein-coated plates and between Exo-depleted FCS and sExo or TEX: s; **c** transwell migration of wt- and ko-MCA cells towards BSA versus 20% FCS; mean % migrating cells±SD (triplicates); significant differences in transwell migration between wt- and ko-MCA tumor cells: *; **d** in vitro wound healing of wt- and ko-MCA cells was evaluated by the scratch assay. After reaching subconfluence, the monolayer was scratched and wound healing was followed microscopically for 48 h–72 h. Representative examples of wt- and ko-MCA cells seeded on coll I-coated plates (wound edge are indicated by a dashed line) and on BSA-, coll I-, coll IV-, LN111-, LN332- or FN-coated plates; the mean % wound area ± SD (3 assays) are shown; the mean % differences in the wound area compared to BSA-coated plates are listed in the table, significant differences are shadowed; **e** transwell migration of wt- and ko-MCA cells towards BSA versus wt-sExo and wt- and ko-TEX was evaluated in Boyden chambers after 16 h of incubation; mean % migrating cells±SD (triplicates); significant differences in migration towards BSA versus sExo and TEX: s; **f** wound healing of ko-MCA cells seeded on BSA-coated plates was evaluated in the presence of medium containing 10% Exo-depleted FCS or wt- and ko-TEX (30 μg/ml) after 24 h; the mean % wound area ± SD (triplicates), significant differences between Exo-depleted FCS versus TEX containing medium: s. Transwell migration and in vitro wound healing of ko-, most strongly dbko-MCA cells is impaired, the difference in wound healing being maintained in matrix protein-coated plates, where distinct to Tspan8ko- and CD151ko-MCA cells, dbko-MCA only migrate on FN-coated plates. Migration is promoted by wt-TEX and, weakly, by Tspan8ko- or CD151ko-TEX in CD151ko-, respectively, Tspan8ko-MCA cells

Transwell migration and migratory activity in the scratch assay (in vitro wound healing) of ko-MCA cells is impaired (Fig. 3c). This accounted for migration on BSA- and matrix protein-coated plates. Migration of wt-MCA was accelerated on coll I-, coll IV-, LN111- and LN332-, but not FN-coated plates. Migration of Tspan8ko- and particularly CD151ko-MCA was less efficiently supported. Dbko-MCA migration became only accelerated on FN-coated plates (Fig. 3d). Only wt-sExo/−TEX supported transwell migration and wound healing, the poor response of dbko-MCA cells indicating additive activities of Tspan8- and CD151-competent TEX as well as additional defects in dbko-MCA tumors (Fig. 3e, f).

Reduced recovery of some adhesion molecules in Tspan8ko- and CD151ko-cells and -TEX (Additional file 1: Figure S1f-h) pointed towards an association with Tspan8 and CD151 and a joint transfer into TEX. Confocal microscopy indicated pronounced CD49f-Tspan8 and CD49f-CD9 colocalization in CD151ko-MCA. But, CD106 did not colocalize with CD9 or Tspan8 in CD151ko-MCA. F-actin preferentially colocalized with Tspan8. In dbko-MCA, colocalization with CD9 was reduced (Fig. 4a). Co-immunoprecipitation confirmed an association of CD49f and CD49c with Tspan8 and CD151 and of CD56 and CD106 with CD151 in cells and TEX. However, after cells were cocultured with wt-TEX, particularly CD151 was recovered in the IP of CD151ko-MCA such that the coimmunoprecipitation pattern lost in selectivity (Fig. 4b).

**Fig. 4:** Adhesion molecule location and association with tetraspanins in wt- and ko-MCA tumor cells. **a** Colocalization of CD49f, CD106 and F-actin (Phalloidin) with CD9, Tspan8 and CD151 was evaluated by confocal microscopy. Representative examples of single staining and overlays are shown (scale bar: 10 μm); **b** coIP of CD49f, CD49c, CD56 and CD106 with CD9, CD151 and Tspan8 in wt- and ko-MCA cells, TEX and wt-TEX-treated cells; **c** WB of wt- and ko-MCA cell lysates after sucrose gradient centrifugation, where the light fractions (1–4) were tested individually and medium dense fractions 5–8 and dense fractions 9–12 were pooled; representative examples are shown and the mean intensity of light fractions (1–4) in comparison to all fractions (3 assays) is shown; significant differences in the recovery in light fractions between wt- and ko-MCA cells: *. CD49f most prominently colocalizes with CD9 and Tspan8 in CD151ko-MCA, whereas CD106 preferentially colocalizes with CD151. F-actin associates with CD9 and Tspan8, but hardly with CD151. CoIP confirmed preferential association of CD49f and CD49c with Tspan8 and of CD56 and CD106 with CD151 in cells and, less pronounced, TEX and wt-TEX-treated cells. In MCA cells, the association of adhesion molecules with tetraspanins is accompanied by pronounced recovery in light density (TEM) fractions

TEM recovery in light density sucrose gradient fractions provides an additional option to control for CD151/Tspan8-adhesion molecule associations. CD49f and CD49c were partially shifted towards heavier fractions in Tspan8ko-, CD151ko- and, more strongly, dbko-MCA cells. Instead, CD56 and CD106 were relocated into heavy fractions only in CD151ko and dbko cells. Both, a Tspan8ko and a CD151ko also, albeit slightly, affected CD9 recovery in light density fractions and, unexpectedly, Tspan8 contributed to CD151 recovery in light density fractions and vice versa (Fig. 4c).

Thus, CD151- and Tspan8-associated adhesion molecules in TEX contribute to migration. In the MCA tumors this relies predominantly on CD49c-, CD49f- and (not shown) CD104-associated Tspan8 and on CD56- and CD106-associated CD151.

### Tspan8 and CD151, invasion and the contribution of TEX proteases

Tetraspanin-associated proteases in cells and TEX contribute to matrix degradation and tissue invasion [57–60]. Wt-TEX strongly degrade collagen IV and LN332 and significantly coll I. FN is not degraded. Whereas degradation of coll I, coll IV and LN332 is partly maintained in single Tspan8ko- and CD151ko-TEX, no degradation is seen with dbko-TEX (Fig. 5a). Zymography confirmed low MMP9 and high MMP2 expression in MCA tumor supernatant, MMP9 recovery being nearly abolished and MMP2 expression strongly reduced in Tspan8ko- and dbko-MCA supernatants (Fig. 5b). Matrigel invasion and penetration of the ko-MCA cells is significantly impaired, with a stronger impact of Tspan8 than CD151 and a more pronounced reduction of dbko-MCA cells (Fig. 5c). Reduced invasiveness of Tspan8ko- and CD151ko-MCA cells is restored by wt- and to some degree by Tspan8ko- and CD151ko-, but not dbko-TEX (Additional file 1: Figure S6a, Fig. 5d).

**Fig. 5:** Invasion of wt- and ko-MCA tumor cells. **a** Wt- and ko-TEX (20 μg/ml) were cocultured with 1 μg matrix proteins for 48 h; matrix protein degradation was evaluated by WB, representative examples are shown; **b** zymography of wt- and ko-MCA culture supernatant collected after 48 h culture in the absence of FCS; MMP9 and MMP2 are indicated; **c** wt- and ko-MCA cells were seeded on matrigel; invasion (crystal-violet staining of matrigel embedded cells) and penetration (counting cells at the lower membrane site after crystal-violet staining) was evaluated after 48 h incubation; representative examples and mean % invading±SD / No of penetrating cells±SD (triplicates) are shown; significant differences in invasion and penetration between wt- and ko-MCA tumor cells: *; **d** ko-MCA cells were seeded on matrigel containing 50 μg/ml TEX. Evaluation was performed as described in (**c**); mean % invading±SD / No of penetrating cells±SD (triplicates) are shown; significant differences in invasion and penetration in TEX-containing matrigel: s. Tspan8ko and dbko TEX poorly degraded coll I, coll IV and LN332 and gelatin. Invasion of Tspan8ko- and/or CD151ko-MCA tumors is severely reduced, but partly rescued by wt-TEX and weakly by Tspan8ko- or CD151ko-TEX; dbko-TEX are ineffective

TEX did not affect protease expression in wt-MCA. Instead, protease expression was rescued by wt- and CD151ko-TEX in Tspan8ko-MCA. Wt-TEX also supported MMP2, MMP3, MMP7, MMP14 and TACE expression in CD151ko-MCA. A weak effect of Tspan8ko-TEX was only seen in membrane-anchored MMP14 and TACE. Dbko-MCA protease expression was upregulated after coculture with wt-TEX. Tspan8ko-TEX only promoted MMP14 expression (Additional file 1: Figure S6b). The strong impact of wt-TEX on dbko-MCA cells may rely on recruitment via MMP14, not being essentially linked to TEM-derived TEX. To control the hypothesis, colocalization of proteases with tetraspanins was evaluated.

Unexpectedly, CD9 colocalizes with MMP2 and TACE in dbko-MCA, but poorly in Tspan8ko- and CD151ko-MCA cells, indicating CD9 taking over compensatory activity in the absence of both Tspan8 and CD151 (Fig. 6a). In wt- and CD151ko-MCA cells MMP2, MMP9, TACE and weakly MMP14 colocalize with Tspan8. CD151 colocalizes with TACE in wt- and Tspan8ko-MCA cells (Fig. 6b). Coimmunoprecipitation of proteases with CD9, Tspan8 and CD151 after mild lysis avoiding TEM complexes disruption confirmed CD9 coimmunoprecipitation with MMP2, MMP9, uPAR and TACE in cells and TEX. Tspan8 and CD151 also coimmunoprecipitated with these proteases, coimmunoprecipitation of uPAR and TACE with Tspan8 and CD151 being stronger in TEX than cells (Fig. 6c). Sucrose gradient fractionation confirmed that in Tspan8ko- and dbko-MCA lysates MMP2 was only recovered in dense fractions and MMP9 was partly shifted to heavier fractions. UPAR and TACE recovery in light fractions was not affected in ko-lysates (Fig. 6d).

**Fig. 6:** Colocalization and coimmunoprecipitation of proteases with tetraspanins in wt- and ko-MCA cells. Confocal microscopy of MMP2, MMP9, MMP14 and TACE with (**a**) CD9 and (**b**) Tspan8 and CD151 in wt- and ko-MCA cells; representative examples of overlays with the indicated proteases and tetraspanins are shown; **c** precipitates of wt- and ko-MCA cell and TEX lysates with anti-MMP2, -MMP9, -uPAR and -TACE were separated by SDS-PAGE, blotting membranes with anti-CD9, -CD151 and -Tspan8; representative examples are shown; **d** lysates of wt- and ko-MCA tumors were fractionated by sucrose gradient centrifugation. After SDS-PAGE of fractions 1–4 and pooled fractions 5–8 and 9–12, membranes were blotted with anti-MMP2, -MMP9, -uPAR and -TACE; representative examples are shown. MMP2, MMP9 and MMP14 preferentially colocalize with Tspan8, TACE colocalizes with Tspan8 and CD151. However, in the absence of Tspan8 and CD151, proteases also associate with CD9, which was confirmed by coIP. Density fractionation indicated impaired invasion being a sequel of the missing association of MMP2 and MMP9 with Tspan8 and/or CD151 in TEM. Recovery of uPAR and TACE in light density fractions being not affected in Tspan8ko- and/or CD151ko-MCA cells points towards TEM-independent associations

We interpret these findings that in MCA cells MMP2 and MMP9 preferentially associate with Tspan8. As Tspan8 expression is weak, only a minor part of proteases is tetraspanin-associated. uPAR and TACE being not shifted to higher density fractions in ko-MCA cells indicates colocalization being (Tspan8- and CD151-)TEM-independent. Nonetheless, by the recruitment of proteases into TEX, wt-TEX strongly promote MCA cell invasion.

In brief, in vitro studies revealed a minor decrease in apoptosis resistance of Tspan8ko- and/or CD151ko-MCA cells due to impaired PI3K/Akt pathway activation. The defect was covered by wt-TEX. Wt-TEX also partially coped with impaired anchorage-independent growth of the ko-MCA lines. There was no evidence for a selective contribution of Tspan8 and CD151 to EMT. Thus, CD151 and Tspan8 are not involved in oncogenesis/oncogenicity of MCA tumors. Instead, a Tspan8ko and a CD151ko affect tumor cell dissemination, which relies on poor recruitment of integrins, CAMs and proteases into TEM / TEM-derived TEX. Tspan8- and CD151-associated molecules are only partly overlapping, accounting for stronger deficits in dbko-MCA. Fittingly, wt- and to a minor degree Tspan8ko- and CD151ko-, but not dbko-TEX suffice for correction. Colocalization and coimmunoprecipitation with CD9 in the absence of Tspan8 or CD151 point towards an engagement of additional tetraspanins, particularly in protease recruitment.

We have not yet taken into account retarded growth start and impaired settlement of wt-MCA in ko-mice. Both features suggest a Tspan8- or CD151-dependent impact of TEX on host cells [61] and a Tspan8- or CD151-dependent contribution of host Exo, which was controlled for BMC and EC.

### Serum exosomes and TEX and hematopoiesis / the premetastatic niche

Ko-MCA settlement in the BM was most strongly impaired in the ko host (Fig. 2c) and TEX can account for tumor progression-associated anemia and immune deviation [62]. A potential impact of Tspan8 and CD151 on hematopoiesis, immunosuppression and metastatic niche preparation was evaluated by coculturing BMC with sExo and TEX. Wt-sExo only corrected for reduced CD44 and CD62P expression in ko-BMC. Instead, BMC responded differently to wt-TEX versus ko-TEX. As far as changes were observed in ALDH1/2 and the progenitor markers CD44, CD62P, TER119, GR1 and CD11b, wt and ko BMC responded alike to wt- and ko-TEX. Instead, KIT and CD34 only responded to wt-TEX and, less pronounced to CD151ko-TEX. We did not see significant differences in hematopoietic growth factors and chemokines. The response to growth factor receptors and chemokine receptors differed depending on TEX and/or the BMC donor. Only wt-TEX suppressed MCSFR expression in wt- and Tspan8ko-BMC. CCR5 expression was reduced in wt- and Tspan8ko-BMC by wt- and Tspan8ko-TEX. CXCR3 expression solely was upregulated by wt-TEX in wt-BMC. CD184 expression became elevated in wt- and CD151ko-BMC by wt-TEX and CD151ko-TEX and in Tspan8ko-BMC by wt-TEX. FOXO3 expression was reduced in wt- and ko-BMC treated with wt-TEX and in wt- and Tspan8ko-BMC cultured with Tspan8ko-TEX (Fig. 7a-c, Additional file 1: Figure S7a-c). We interpret these findings that the impact of TEX on progenitor promotion or suppression is Tspan8- and CD151-independent, whereas FOXO3 and hematopoietic receptor modulation apparently relies on cooperation with Tspan8 or CD151, which was controlled by co-immunoprecipitation of FOXO3, KIT, MCSFR, CD184, TER119 and CD11b with CD9, Tspan8 and CD151. TER119 and CD11b only coimmunoprecipitated with CD9. Instead, KIT, MCSFR, CD184 and the transcription factor FOXO3, abundantly expressed in BMC [63], also coimmunoprecipitated with Tspan8 and CD151, coimmunoprecipitation being not significantly altered by wt-TEX treatment (Fig. 7d).

**Fig. 7:** The impact of Tspan8 and CD151 on hematopoiesis. The impact of Tspan8 and/or CD151 on hematopoietic cells and hematopoietic cell modulation by wt-sExo or -TEX was evaluated in vitro using freshly harvested BMC, cultured for 48 h–72 h with sExo and TEX. **a-c** Flow-cytometry analysis of tetraspanins, progenitor markers, growth factors and receptors, chemokines and receptors andFOXO3 after culture with wt-sExo or wt- and ko-TEX; mean values of triplicates are shown, significant differences by coculture with wt-sExo are indicated by s (grey), by coculture with wt- and ko-TEX by s (black), by coculture with wt-TEX by σ; **d** Untreated and wt-TEX-treated wt- and ko-BMC lysates were precipitated with FOXO3, KIT, MCSFR, CD184, TER119 and CD11b and blotted with anti-CD9, -CD151 and -Tspan8. Wt-sExo rescued CD44 and CD62P expression in ko-BMC. Wt- and ko-TEX provoked a slight reduction of ALDH1+, the megakaryocyte marker CD62P and the erythroid progenitor marker TER119 and promoted myeloid progenitor expansion, indicating that these effects were Tspan8- and CD151-independent; altered cytokine and receptor expression was mostly restricted to wt-TEX treatment. Receptors and FOXO3 coimmunoprecipitated with Tspan8 and CD151. Only CD9 coimmunoprecipitated with TER119 and CD11b. The association of Tspan8 and CD151 with RTK and GPCR might support homing and settling of MCA in the BM

Thus, reduced CD34, KIT and ALDH1/2 expression in ko-BMC could indicate a minor contribution of Tspan8 and CD151 to early hematopoiesis. Impaired thrombopoiesis and erythropoiesis becomes aggravated Tspan8- and CD151-independent by TEX. This also accounts for expansion of CD11b + BMC. Reduced expression of CD44 and CD62P, a megakaryocyte and endothelial cell marker, corrected by wt-sExo, could contribute to impaired MCA homing into the BM, reduced TER119 expression may account for tumor-associated anemia. The TEX-promoted CD11b upregulation in wt- and ko-BMC likely is associated with a shift towards MDSC or tumor growth-promoting M2 Mϕ. The reduced recovery of Kit+ and CD34+ cells in all ko BMC and coimmunoprecipitation of KIT, MCSFR, CD184 and FOXO3 with Tspan8 and CD151 point towards Tspan8 and CD151 supporting receptor-promoted hematopoietic cell activation.

### The impact of serum-Exo and TEX on angiogenesis

A contribution of sExo and TEX tetraspanins to angiogenesis [64] was evaluated using EC-enriched cultures from wt- and ko-lungs. EC tetraspanin expression is not significantly affected by sExo or TEX. But, wt-TEX promoted CD31 and CD34 expression in wt- and ko-EC, CD144 in Tspan8ko-EC and CD106 and CD62P in CD151ko-EC. Wt-TEX also promoted OPN, SDF1, VEGFR2, FGFR3, EphA4 and CD184 in wt- and ko-EC and wt-sExo sufficed for upregulation of OPN, VEGFR2 and EphA4 in ko-EC (Fig. 8a). Controlling for angiogenic receptor expression in MCA cells confirmed VEGFR2, VEGFR3 and EphA4 upregulation by wt-TEX and correction in ko-MCA by wt-sExo. Lyve expression was only promoted in CD151ko-MCA by wt-sExo and -TEX (Fig. 8b).

**Fig. 8:** Tspan8, CD151 and angiogenesis in ko mice and ko MCA tumors. Dispersed lung cells were cultured for 3wk-4wk to enrich and expand EC. EC were cocultured with wt-sExo or wt- and ko-TEX for 48 h–72 h. **a** EC flow-cytometry analysis of tetraspanins, EC markers, chemokines and angiogenic receptors including representative examples and (**b**) of MCA angiogenic receptor; **a,b** mean % stained cells (3 assays), significant differences between wt- and ko-EC or -MCA cells: *, significant differences by coculture with sExo: s (grey) or TEX: s (black); **c-e** confocal microscopy of wt-, Tspan8ko-, and CD151ko-EC cultured in the absence or presence of wt-sExo or -TEX and stained with anti-Tspan8 or anti-CD151 and counterstained with (**c**) anti-CD184, **d** anti-EphB4, **e** anti-VEGFR2, single staining and overlays are shown (scale bar: 10 μm); **f** untreated and wt-TEX-treated wt- and ko-MCA lysates were precipitated with anti-VEGFR2, -VEGFR3, -FGFR3 and EphA4. Dissolved precipitates were blotted with anti-Tspan8 or anti-CD151. Representative WB examples are shown. Ko-EC express CD31, CD34, OPN, VEGFR2, and EphA4 at a reduced level; in CD151ko-EC additionally CD106 and CD62P expression is reduced. Wt-sExo promote OPN, VEGFR2 and EphA4 expression in ko-EC; wt-TEX activate EC marker, OPN, SDF1, VEGFR2, EphA4 and CD184 expression in wt- and ko-EC. In ko-MCA cells, wt-sExo and -TEX support VEGFR2, VEGFR3 and EphA4 expression. Upregulated expression, accompanied by colocalization and coimmunoprecipitation, might well account for Tspan8- and CD151-TEX promoted EC activation

Confocal microscopy accredited pronounced CD184 colocalization with Tspan8 and CD151 in wt-sExo-treated CD151ko- and Tspan8ko-EC. Wt-TEX also promoted pronounced CD184 colocalization with Tspan8 and CD151 in wt-EC (Fig. 8c). Similar findings accounted for EphA4 and VEGFR2, although the impact of sExo and TEX was weaker due to colocalization also in the absence of sExo or TEX (Fig. 8d, e).

Evaluating the impact of sExo and TEX on expression and colocalization of VEGFR3 in wt-, Tspan8ko- and CD151ko-MCA indicated strong colocalization with Tspan8 in TEX-treated wt- and CD151ko-MCA, but less pronounced with CD151 in Tspan8ko-MCA, suggesting preferential colocalization of VEGFR3 with Tspan8 (data not shown). CoIP of VEGFR2, VEGFR3, FGFR3 and EphA4 with CD151 and Tspan8 in MCA-lysates confirmed VEGFR2 preferentially associating with CD151, and VEGFR3 with Tspan8. EphA4 and FGFR3 associate with both. Notably, in most instances, coimmunoprecipitation is stronger after coculture with wt-TEX (Fig. 8f).

These analyses revealed defects in angiogenesis being partly host- and partly tumor-related. Defects in RTK expression can mostly be rescued by TEX, sExo are more efficient in stimulating angiogenic factor expression. The increased recovery of Tspan8 and CD151 in wt-sExo- or -TEX-treated ko cells was unexpected and might indicate a direct transfer from sExo/TEX into the tumor cell, which requires further exploration.

Tspan8ko-, CD151ko- and dbko-MCA tumors poorly disseminate in the autochthonous host, which relies on the contribution of Tspan8 and CD151 to TEX biogenesis particularly the recruitment of associated proteins that account for adhesion, migration, invasion and (lymph)angiogenesis. Mitigated defects in ko tumor cell dissemination grown in wt-mice are based on the support of angiogenesis by host Exo.

## Discussion

There is ample evidence for the importance of TEX in tumor progression and angiogenesis [65] with a suggested feedback by host-derived Exo. We approached the topic using Tspan8ko and/or CD151ko hosts and MCA tumors, based on the following considerations. First, tetraspanins act as molecular facilitators by associating with a multitude of proteins that become assembled in special glycolipid-enriched membrane domains, TEM [17, 66, 67]. Second, tetraspanins are engaged in Exo biogenesis such that the complete armament of TEM is transferred into Exo [43]. Third, tetraspanin complexes contribute to target binding and uptake [15]. Fourth, both Tspan8 and CD151 promote angiogenesis and tumor progression [21, 41, 68–70]. Last, there are hints that CD151 and Tspan8 may use different partners and pathways to achieve alike effects [21].

The model confirmed metastasis-promotion of Tspan8 and CD151 as well as a host Tspan8 / CD151 contribution. Wt MCA tumors poorly disseminate in Tspan8ko and/or CD151ko hosts and Tspan8ko- and/or CD151ko-MCA poorly disseminate in the autochthonous host, whereas dissemination is enhanced in the wt host. We will discuss our interpretations after outlining the limits of the experimental system.

### Strengths and limitations of the Tspan8ko / CD151ko criss-cross model

The potency of the model, outlined above, also accounts for the MCA tumors, though CD151 expression was not high and Tspan8 expression was low. Nonetheless, Tspan8- and CD151 were enriched in Exo compared to parental cells [9].

However, interpretations need to take into account some limitations. First, cells deliver different types of Exo [7, 9, 13, 71]. To incorporate this aspect, purified Exo would have to be sorted according to selective markers of caveolae-, raft-, lipid- and GOLGI-derived Exo. Due to a shortage of selective markers, separating exclusively TEM-derived Exo was technically not feasible. In addition, tetraspanins are not exclusively located in TEM and the tetraspanin composition in individual TEM / TEM-derived Exo varies [72]. As all types of Exo share lipid-ordered membranes, working with a pool of Exo prohibited controlling coimmunoprecipitation after mild lysis by density distribution. To take this into account, cell lysate proteins recovered at a different density from TEM-located tetraspanins were considered as not being TEM-derived. For a third, model-related phenomenon, two interpretations cannot be mutually excluded. A high number of proteins colocalizes and coimmunoprecipitates with CD9, colocalization / coimmunoprecipitation being frequently, but not consistently stronger in Tspan8ko or CD151ko cells. In the latter case, replacement of Tspan8 / CD151 by CD9 could be envisaged. Alternatively, by the high abundance of CD9 compared to CD151 and Tspan8, CD9-TEM and CD9-TEM-derived Exo may be dominating.

In brief, working with a pool of Exo prohibits an unequivocal assignment to Tspan8, CD151 or additional tetraspanins, particularly CD9. Thus, with few exceptions, the suggestion of divergent/additive activities of Exo Tspan8 and CD151 are based on different effects seen inTspan8ko and CD151ko cells and on stronger effects in dbko than Tspan8ko or CD151ko cells and Exo.

### Tspan8, CD151 and Tspan8-/CD151-complexes in tumor progression

Distinct to epithelial cancer induction in CD151ko mice [73], MCA tumor induction was not affected by a deficit in Tspan8 or CD151 [41]. No major changes in common tumor markers being observed, the more rapid local growth of a dbko-MCA tumor fortifies this suggestion. CD151 is not essentially linked to tumor induction. Nonetheless, CD151 may contribute to oncogenesis in epithelial tumors via the crosstalk with a surrounding that promotes integrin activation initiating either FAK and downstream signaling or RTK activation [29, 74–78].

On the other hand, a Tspan8ko and a CD151ko affected anchorage-independent growth, which was partially rescued by wt-TEX. Anoikis execution, initiated via perturbation of mitochondria or death receptor activation, proceeds via activation of caspases and downstream pathways with activation of endonucleases and DNA fragmentation. Anoikis resistance being vital for tumor progression and metastasis formation, tumor cells use several pathways to circumvent anoikis. A shift towards anoikis-protecting integrins was not observed (79), only in CD151ko/dbko MCA CD151 expression was reduced and rescued in wt and Tspan8ko mice. Adhesion to the ECM can promote FAK, Src and ILK activation which promote PI3K/Akt and MAPK pathway activation (79), seen in Tspan8kd and CD151kd pancreatic adenocarcinoma (40), but not in the ko MCA. Alternatively, integrins mediate growth factor receptor activation [79, 80]. Though EGFR and MET expression were not affected, expression of several RTK including TGFβR, VEGFR2 and EphA4 were reduced in Tspan8ko and/or CD151ko MCA, which could have added to reduced apoptosis resistance. Finally, EMT contributes to anoikis resistance [79, 81], the EMT phenotype being accompanied by a reduction of E-cadherins / β-catenin, upregulation of the mesenchymal markers vimentin and FN and MMP activation. Central for EMT induction are the transcription factors Snail, ZEB1/2, Twist, NFκB and HIF [79, 82].We only noted a slight reduction of vimentin in Tspan8ko and CD151ko MCA and a reduction in FN expression, stronger in CD151ko- than Tspan8ko-MCA. Wt-TEX merely sufficed for a significant rescue of FN in Tspan8ko MCA. Expression of the central EMT-related transcription factors was not affected by the Tspan8ko and/or CD151ko and remained stable in the presence of wt-TEX. Instead, expression of Nanog and NOTCH that can contribute to EMT [83, 84] was reduced in Tspan8ko and CD151ko MCA and was rescued by wt- and ko-TEX. The latter suggests Tspan8- and CD151-independent TEX components accounting for the rescue.

In brief, Tspan8 and CD151 do not significantly contribute to drug resistant, only proliferation of the dbko-MCA line being more sensitive to cisplatin treatment. As PI3K/Akt pathway activation (data not shown) and pBAD and BclXl expression were reduced in Tspan8ko- and dbko-MCA cells and corrected by wt-TEX, mitigated PI3K/Akt activation likely sufficed for impaired proliferation, but not for affecting mitochondrial integrity or promoting DNA degradation. Also excluding a major contribution of MCA Tspan8 and CD151 to EMT, a rescue of NOTCH and Nanog by TEX being Tspan8- and CD151-independent, we suggest reduced anchorage-independent growth of Tspan8ko and CD151ko MCA to rely on multiple factors that partly are Tspan8- and CD151-independent.

Poor migration of Tspan8ko- and CD151ko-tumors on collagen I, collagen IV, LN111 and LN332 is due to distorted CD49c-Tspan8 and CD56- and CD106-CD151 cooperation, expression of these adhesion molecules being slightly reduced in ko-MCA cells and TEX. However, CD49c and CD49f, preferred LN-binding integrin partners of CD151 and Tspan8 [40, 85–87], also precipitated with CD9 in the absence of Tspan8 and/or CD151. A contribution of CD9 to migration [88–90] was suggested to rely on clustering associated adhesion molecules and concomitantly reducing TACE activation [91]. However, although CD49c and CD9 shifted to heavier fractions particularly in dbko cell lysates, in wt lysates, too, a higher proportion of CD9 than of Tspan8 and CD151 was recovered in heavier fractions. We interpret the finding indicating CD9 being only partly located in TEM. Accordingly, TEX CD9-integrin complexes might differ from TEM-derived complexes. Whether non-TEM CD9-integrin complexes substitute for Tspan8 and CD151 or account for distinct adhesion, remains to be answered. Only dbko MCA showing pronounced migration on FN-coated plates suggests an engagement of CD9-associated integrins. However, depending on the integrin profile, CD9 may also inhibit FN binding [92].

CD56 and CD106 selectively coimmunoprecipitated with CD151. In cancer, CD151 and CD56 / CD106 are jointly upregulated [93, 94], CD106 upregulation proceeding via the impact of CD151 on MET signaling [94], CD151-dependent activation of MET signaling in promoting motility being also described for EC [94], and a CD151-CD49c or -CD49f complex promotes motility of breast cancer cells via MET activation [74], which may also account for CD56. Notably, the selective shift of CD56 and CD106 towards heavier sucrose gradient fractions in CD151ko and dbko cells indicates that CD151 and Tspan8 are partly recovered in distinct TEM domains and, accordingly, will be separately recruited into EE / TEX.

Tspan8 and CD151 also distinctly contribute to invasion. Tspan8ko- and CD151ko-MCA are poorly invasive, matrigel penetration of dbko-MCA being further reduced. Coculture of Tspan8ko- and CD151ko-MCA cells with wt- and ko-TEX confirmed strongly reduced efficacy of ko-TEX in restoring invasiveness compared to wt-TEX. This relies on the association of Tspan8 and CD151 with proteases. MMP2 and MMP9 are most strongly reduced in Tspan8ko-TEX, recovery of the membrane-anchored proteases TACE, ADAM10 and MMP14 is more severely affected in CD151ko-TEX. Sucrose gradient fractionation indicated a shift of MMP2 and MMP9 to heavier fractions in Tspan8ko-, but not of uPAR and TACE in CD151ko-lysates, indicating CD151 associating with uPAR and ADAM10 preferentially in Non-TEM internalization domains. The GPI-anchored uPAR can associate with IGF2R (insulin like growth factor 2 receptor), which promotes internalization [95]. uPAR also associates with LRP-1 (LDL receptor related protein 1), which recruits VEGFR2 and fosters internalization upon ligand binding [96]. Furthermore, cathepsin B and uPAR were described to regulate LN332-bound CD151-CD49c/CD29 complex expression in glioma, the components of this multimeric complex coimmunoprecipitating [97]. Downregulation of cathepsin B or uPAR is accompanied by reduced CD151 and CD49c/CD29 expression and downstream FAK, src and paxillin phosphorylation [97]. TACE is partly recovered in TEM [98] and coimmunoprecipitates with CD151. It was described that palmitoylated Tspan12 associates with ADAM10, enhances ADAM10 prodomain maturation and amyloid precursor protein shedding [99]. We noted coimmunoprecipitation of CD151 with TACE, the major sheddase for tumor necrosis factor α (TNFα), EGFR ligands, CD62L and the IL6R [100]. Opposing expectation, uPAR and TACE were not shifted to heavier density fractions in CD151ko MCA. Thus, uPAR and TACE recruitment into TEX may not proceed via internalized TEM. Irrespective of TEX recruitment, the findings are in line with protease upregulation/activation relying on tetraspanin-associations, where activation of integrins and RTK can drive protease expression [22, 44, 101, 102].

Taken together, Tspan8 and CD151 not significantly contributing to apoptosis resistance and EMT of MCA tumors argues against an involvement in oncogenicity. However, Tspan8 and CD151 support migration and invasion, which relies on clustering adhesion molecules and proteases in invagination prone membrane domains, fostering release in TEX. Tspan8 preferably associates with integrins, MMP2 and MMP9; CD151 primarily cooperates with CAMs and membrane-anchored proteases, which accounts for the additive defects in dbko-MCA. Delivery of distinct TEX, only part of them being TEM-derived and/or harvesting Tspan8 and CD151 explains the gradual rather than on/off effects of Tspan8 and CD151 deletion.

### Tspan8, CD151 and the crosstalk between tumor and host

Impaired settlement of Tspan8ko- and CD151ko-MCA in the autochthonous BM, partly restored in the wt-host, suggested a contribution of sExo/TEX-Tspan8 and -CD151 to tumor cell settlement in the BM [103, 104] and to deviation of hematopoiesis [53, 105].

A slight reduction of CD9, CD63 and early hematopoietic progenitors (KIT+, CD34+) in Tspan8ko- and CD151ko-BMC was not corrected or aggravated by coculture with wt-sExo or wt-TEX. We interpret the reduced recovery of CD9, CD63 and KIT in ko mice indicating a contribution of Tspan8 and CD151 to early hematopoiesis maintenance as described for CD9 and CD63 in embryonic development [61, 106]. Not yet answered for Tspan8 and CD151, this suggestion requires follow-up studies. Furthermore, CD9 and CD151 are engaged in thrombopoiesis, CD9 also affects myelopoiesis and CD151 erythropoiesis. These activities essentially depend on the association with integrins and include the crosstalk with the ECM and mesenchymal stem cells [107–111]. We noted reduced CD62P, TER119 and GR1 expression in Tspan8ko and CD151ko BMC. With the exception of CD62P and CD44 (only CD151ko), these defects were not corrected by wt-sExo. Instead, wt- and ko-TEX promoted a further reduction of Ter119, CD62P and an expansion of CD11b. Thus, the impact of TEX on deviation of committed hematopoietic progenitors is Tspan8- and CD151-independent. On the other hand, reduced expression of FOXO3, the central transcription factor in hematopoiesis [112], and KIT, MCSFR and CD184 receptors were mostly affected by wt-, but not by ko-TEX. These molecules coimmunoprecipitate with CD151 and Tspan8, implying the Tspan8- or CD151-associations assisting expression/activation. The finding strengthens the importance of the interplay between tetraspanins and receptor kinases also in non-transformed cells. Finally, wt-sExo may well contribute to MCA settlement in the BM by promoting adhesion- and homing-facilitating higher CD62P and CD44 expression [113, 114]. Wt-TEX can support this process by CD184 induction, possibly in concert with additional chemokine receptors [115, 116]. A direct contribution to CD184 expression was described for CD9, CD184 upregulation modulating megakaryocyte motility and leukemia dissemination [107, 117]. Furthermore, a CD63 mutant inhibits HIV1 entry by disrupting the trafficking of CD184 to the plasma membrane [118]. Though the engagement of tetraspanins in GPCR activation is not fully elucidated, GPCR engagement in membrane lipid microdomains / rafts and Exo contributes to the dynamic of intercellular communication including cytoskeleton arrangement and signaling [119–121], where coimmunoprecipitation points towards Tspan8 and CD151 contributing to CD184-promoted homing and settlement of MCA tumor cells within the BM environment.

In brief, a suggested contribution of Tspan8 and CD151 to early hematopoiesis requires further exploration. TEX-promoted impaired erythropoiesis, thrombopoiesis and immune deviation relies not or only partly on Tspan8 and CD151. However, Exo/TEX Tspan8 and CD151 assist hematopoiesis maintenance by growth factor receptor stabilization and tumor cell homing by adhesion molecule clustering and chemokine receptor upregulation.

Tspan8ko- and CD151ko-EC revealed defects in OPN [122], VEGFR2 [123] and EphA4 [124] expression. CD151ko-EC additionally showed reduced CD106 and CD62P expression [68, 125, 126]. These defects were not only coped by wt-TEX, but expression of CD31, CD34, CD62P, OPN, SDF1, VEGFR2, VEGFR3, FGFR3, EphA4 and CD184 was stimulated. Wt-sExo supported OPN, SDF1, VEGFR2 and EphA4 upregulation. Similar “corrections” being not seen after coculture with dbko-TEX and rarely with Tspan8ko- or CD151ko-TEX (data not shown) confirms the share of sExo/TEX-Tspan8 and -CD151 to angiogenesis. The contribution of tetraspanin microdomains via the association with e.g. CD54, CD106 and CD62P on EC was repeatedly described [68]. Thus, CD63, CD82 and CD151 bridge VEGFR2 on EC via CD29, which initiates via downstream signaling the response to VEGF [127, 128]. CD9 in association with CD29 and CD61 also promotes EC migration [129] and EWI-F (CD9P-1) inhibits angiogenesis by downregulation of CD151 and CD9 [130], the contribution of CD151 also relying on its palmitoylation, which stimulates PI3K/Akt and MAPK signaling [131]. Furthermore, CD9 promotes angiogenesis in response to fibroblast growth factor (FGF) by linking JAM to CD51/CD61-initiated signaling [132] and CD151 fosters angiogenesis on LN substrates, Akt, e-NOS, Rac and Cdc42 becoming activated via CD151-associated integrins [133]. In addition, CD151 can promote EC proliferation, migration and tube formation by stimulating MET signaling [94]. Also and of special interest, CD151-CD49f/CD29 complexes instruct embryonic stem cells towards differentiation into EC [31]. Tspan8 TEX-induced angiogenesis is accompanied by upregulation of Tspan8, von Willebrand factor (vWF), CXCL5, macrophage migration inhibitory factor (MIF) and CCR1 in EC. Coculture with Tspan8-CD49d TEX promotes EC proliferation and sprouting and EC progenitor maturation [39, 70]. Previous studies in Tspan8ko and CD151ko mice confirmed impaired angiogenesis and suggested a contribution due to adhesion molecules not being assembled in Tspan8ko and CD151ko TEM, which resulted in impaired adhesion and migration [41]. Notably, tetraspanin webs are also engaged in lymphangiogenesis. CD9 promotes lymphangiogenesis by a linkage to VEGFR3 via CD49e or integrin α9 [47]. Lymphangiogenesis induction in prostate cancer essentially depends on high CD151 expression [45].

Taken together, CD9, Tspan8 and CD151 contribute to EC/lymphatic EC activation, proliferation and tube formation. This relies in part on direct activation via palmitoylated tetraspanins, but mostly on cellular or matrix protein ligation of associated CAMs, selectins and integrins, which in turn account for angiogenic receptor recruitment and internalization-promoted activation. Due to the recruitment of TEM microdomains into Exo, deficits of Tspan8ko and CD151ko EC can mostly be balanced by sExo, whereas TEX fortify (lymph)angiogenesis.

Finally, Tspan8 and CD151 assist angiogenic receptor expression in MCA tumor cells and TEX, VEGFR2 [127, 128] being reduced in Tspan8ko and CD151ko, VEGFR3 [41, 45, 47, 48] and EphA4 [124] being more strongly reduced in Tspan8ko- and dbko-MCA. VEGFR2, EphA4 and Lyve are rescued by wt-sExo and wt-TEX [134], VEGFR3 is rescued by wt-TEX. The angiogenesis-related receptors colocalize in EC and coimmunoprecipitate in MCA with Tspan8 (preferentially VEGFR3) and CD151 (especially VEGFR2). Coimmunoprecipitation being strengthened after coculture with TEX is in line with the cooperation of tetraspanins with RTK [135–137]. The contribution of Ephrin receptors relies on acting as a hub for internalization and activation of RTK [138, 139], a connection to tetraspanins being described for the entry of hepatitis C virus into liver cells, where uptake by a CD81-claudin1 complex is facilitated by EphA2 that supports internalization and activation of the EGFR [140].

Deficits in angiogenic receptor expression in Tspan8ko and CD151ko MCA being partly corrected by wt-sExo and more efficiently wt-TEX suggests that tetraspanin-promoted RTK upregulation in MCA tumors proceeds like in EC via tetraspanin-associated adhesion molecules. The tetraspanin-integrin-RTK complex being transferred into TEX, both binding- and uptake-initiated target activations are conceivable.

## Conclusion

The criss-cross evaluation of wt, Tspan8ko, CD151ko and dbko MCA tumor and host cells confirmed tumor- and host-derived Tspan8 and CD151 additively assisting metastasis, defects in cooperation with adhesion molecules, proteases, RTK and GPCR being only partly overlapping. However, due to wt-sExo and wt-TEX being not sorted according to their origin from Tspan8 or CD151 TEM, the distinct contributions of Tspan8 versus CD151 to tumor progression occasionally became veiled in Exo. Nonetheless, we could demonstrate metastasis-promoting Tspan8 and CD151 activities to proceed at multiple levels due to Tspan8 and CD151 cooperating with different partners in distinct cell populations. Support of tumor cell migration and invasion is based on adhesion molecule and protease associations. The tetraspanin-adhesion molecule and -protease complexes being transferred into TEX, wt-TEX treatment copes with ko-MCA deficits. TEX-promoted deviation of hematopoietic progenitor maturation relies not or merely to a minor extent on Tspan8 or CD151. Instead, wt-TEX facilitate MCA recruitment and settlement in the BM by associating with adhesion molecules and chemokine receptors. Angiogenesis mostly affected in CD151ko- and lymphangiogenesis in Tspan8ko-MCA and -EC is reestablished by sExo and boosted by TEX, activation of GPCR and RTK via tetraspanin-associated adhesion molecules being of central importance.

The common theme is the “facilitator” role of tetraspanins [141] and the engagement of TEM in Exo-biogenesis and -binding [142]. Though open questions remain, the poor responsiveness of dbko-MCA suggests a joint blockade of Tspan8 and CD151 efficiently hampering several exosome-provided prerequisites for tumor progression.

## Additional file

Additional file 1: **Table S1.** Primers. **Table S2.** Reagents. **Figure S1.** Characterization of MCA tumors, bone marrow cells and endothelial cells from Tspan8ko- and/or CD151ko-mice. **Figure S2.** Tspan8- and CD151-dependence of TEX and sExo delivery and uptake. **Figure S3.** Ex vivo analysis of tetraspanin, adhesion molecule and angiogenic factor expression in MCA tumors. **Figure S4.** TEX and apoptosis resistance of wt- and ko-MCA tumor cells. **Figure S5.** The impact of TEX on EMT. **Figure S6.** TEX proteases and invasion of Tspan8ko and/or CD151ko MCA cells. **Figure S7** Flow-cytometry examples on the impact of sExo and TEX uptake on BMC subpopulations. (PDF 4883 kb)

## Abbreviations

BMC: Bone marrow cells
coll: Collagen
dbko: Tspan8ko/CD151ko
EC: Endothelial cells
ECM: Extracellular matrix
EE: Early endosomes
Exo: Exosomes
FAK: Focal adhesion kinase
FGF: Fibroblast growth factor
FITC: Fluorescence isothiocyanate
FN: Fibronectin
GPCR: G-protein-coupled receptor
GPI: Glycosylphosphatidylinositol
HGF: Hepatocyte growth factor
IP: Immunoprecipitation
kd: Knockdown
ko: Knockout
LB: Latex beads
LN: Laminin
LNC: Lymph node cells
LRP: Low density lipoprotein receptor-related protein
MCA: Methylcholanthrene
MCSFR: Macrophage colony stimulating factor receptor
MDSC: Myeloid-derived suppressor cells
MIF: Macrophage migration inhibitory factor
MMP: Metalloproteinase
MVB: Multivesicular bodies
OPN: Osteopontin
PBL: Peripheral blood leukocytes
RTK: Receptor tyrosine kinase
sc: Subcutaneously
sExo: Serum-Exo
TEM: Tetraspanin-enriched membrane microdomains
TEX: Tumor exosomes
TF: Tissue factor
ThbSp: Thrombospondin
TNF: Tumor necrosis factor
VEGF: Vascular endothelial growth factor
vWF: Von Willebrand factor
WB: Western blot
wt: Wild type
